# Computational Intelligence Method for Detection of White Blood Cells Using Hybrid of Convolutional Deep Learning and SIFT

**DOI:** 10.1155/2022/9934144

**Published:** 2022-01-12

**Authors:** Mohammad Manthouri, Zhila Aghajari, Sheida Safary

**Affiliations:** ^1^Electrical and Electronic Engineering Department, Shahed University, Tehran, Iran; ^2^Khaje Nasir University of Technology, Electronic and Computer Engineering Faculty, Tehran, Iran; ^3^Department of Computer Engineering, Islamic Azad University North Tehran Branch, Tehran, Iran

## Abstract

Infection diseases are among the top global issues with negative impacts on health, economy, and society as a whole. One of the most effective ways to detect these diseases is done by analysing the microscopic images of blood cells. Artificial intelligence (AI) techniques are now widely used to detect these blood cells and explore their structures. In recent years, deep learning architectures have been utilized as they are powerful tools for big data analysis. In this work, we are presenting a deep neural network for processing of microscopic images of blood cells. Processing these images is particularly important as white blood cells and their structures are being used to diagnose different diseases. In this research, we design and implement a reliable processing system for blood samples and classify five different types of white blood cells in microscopic images. We use the Gram-Schmidt algorithm for segmentation purposes. For the classification of different types of white blood cells, we combine Scale-Invariant Feature Transform (SIFT) feature detection technique with a deep convolutional neural network. To evaluate our work, we tested our method on LISC and WBCis databases. We achieved 95.84% and 97.33% accuracy of segmentation for these data sets, respectively. Our work illustrates that deep learning models can be promising in designing and developing a reliable system for microscopic image processing.

## 1. Introduction

Despite decades of efforts and research in controlling infection diseases, they are still among the most challenging issues in public health. According to the World Health Organization (WHO), infectious diseases are now the world's most deadly communicable disease and are ranked as the 4th leading cause of human death. They are among the top global problems with human, social, and economic impacts across the globe. Therefore, the development of robust systems for early diagnosis and investigating the source of the epidemic are critical to address this global, life-threatening issue.

One important part of the body's immune system is white blood cells (WBC). The white blood cells protect the body against infectious diseases. There are five different types of white blood cells, named as lymphocytes, monocytes, eosinophils, basophils, and neutrophil. The number of white blood cells, as well as their structure, is important in the diagnosis of different infection diseases, such as HIV, rubeola, poliovirus, and chickenpox [1, 2]. This test, named as hemogram test, is done by evaluating the blood cells under a microscope. However, due to the different types of white blood cells and their complex structures, the study of blood vessels manually is highly prone to error [3]. Therefore, a lot of researchers have explored different techniques to help with automatic detection of white blood cells with high accuracy accurately.

In recent years, researchers have investigated and proposed different computational intelligence techniques for infection diseases diagnosis. These techniques include but not limited to transfer learning and deep learning [4–6]. Many researchers have focused on using these computational techniques to detect the white blood cells due to their importance in diagnosing a variety of infectious diseases. Most of these studies have focused on classification and segmentation of the white blood cells. Given the importance of detecting white blood cells, in this paper, we will first review the prior literature on classification and segmentation of the white blood cells. We will present a deep learning method using convolutional neural networks to improve the prior studies. One of our motivations to use convolutional neural networks is because they do not require seeing the entire object. Therefore, it can be a good choice to deal with cells at the edge of the microscopic images as well. We use the Gram-Schmidt algorithm to segment the nuclei in the peripheral blood samples. Next, we use Scale-Invariant Feature Transform (SIFT) feature detection to extract the most predictable features. To keep spatial neighbourhood dependences, which are specifically important in processing image data, we will use convolutional neural networks to learn contextual dependencies. For the classification purpose, we use the weighted two-phase test sample sparse representation method (WTPTSSR) that is an improvement of the method two-phase test sample representation (TPTSR) method [7]. Our motivation to choose WTPTSSR over TPTSR is that this approach keeps the locality information. Therefore, it could be more appropriate for the image classification context.

The rest of this paper is organized as follows. In Section 2, we will review the different techniques that have been used for image segmentation and classification. In Section 3, we will describe our proposed method in two parts. First, we will explain the segmentation and classification steps in detail. Following that, the simulation experiments of segmentation and classification phases will be discussed in Section 4. Next, we will describe our experiments and will report the results of our proposed method. Eventually, we will provide a discussion on how our approach provides insights in detecting white blood cells and how our method can be further improved by future research.

## 2. Related Work

The diversities of the white blood cells make their detection very challenging. Many researchers have investigated different techniques in this domain. These studies mostly relied on image classification and segmentation to detect the white blood cells and investigate their structures. Otsu's thresholding method is used recurrently in the circular histogram to segment the white blood cells [8] by Wu et al. In this paper, Otsu's method is applied to components H and S of the HSI color model. Gautam and Bhadauria improved the contrast of the blood microscopic image and used Otsu's thresholding for the segmentation of the white cell nucleus [9]. Mohapatra et al. did the preprocessing step by applying the median filter on the images in order to eliminate possible noises and used *K*-means clustering in the Lab color model to divide pixels of the blood microscopic images [10]. *K*-means clustering and the Lab color model for segmentation of the white cells nuclei have been also explored [11, 12]. Theera-Umpon used *c*-means fuzzy clustering and morphological operators to segment white cell nuclei [13]. Pan et al. used ELM classifications to extract white blood cells via utilizing visual simulations [14]. They demonstrated that ELM has equivalent performance compared to the SVM and can find efficient samples actively and train the classification model in real time, without the need to adjust the parameters.

Ko et al. [15] provided a step-by-step integration method for nucleus segmentation based on the mean-shift clustering. They also used GVF (extreme learning machine) active curve to segment the cells' cytoplasm. Hamghalam et al. used a combination of Otsu's thresholding method and a snake method-based active curve to segment the nucleus and the cytoplasm in the white blood cells [16]. Rezatofighi et al. proposed a new method for the segmentation of white blood cell nuclei based on Gram-Schmidt orthogonality [17]. They further improved their work by proposing an active curve for cytoplasmic segmentation [18].

For microscopic image edge detection, Nakib et al. [19] used a microcanonical annealing approach to optimize their criterion function through benchmarking two-dimensional exponential entropy. In [20], genetic algorithms and wavelet were used to automatically estimate the number of thresholds for multilevel thresholding of the histogram. They examined their approach of different images, including microscopic blood images. The detection process is designed to detect the ovals in blood images and extract the best of the ovals with DE algorithm. They used the Gram-Schmidt orthogonality algorithm to segment the white blood cells. In order to characterize and extract the types of white blood cells, which could have five different types, the SIFT algorithm and deep convolutional neural network were used. The deep convolutional neural network they used consists of three layers of convolution and two full layers of pooling. To address the small data size, they used WTPTSSR algorithm [21].

## 3. The Proposed Method

In this section, we will first outline the segmentation process, which is primarily based on Gram-Schmidt orthogonality. We will then do the classification process, using Scale-Invariant Feature Transform (SIFT) feature detection and convolutional deep neural network.

### 3.1. Segmentation

We used Gram-Schmidt orthogonality to segment the nuclei in the peripheral blood samples. To do that, we first extracted a three-dimensional vector for each pixel based on their RGB components. Subsequently, the weight vector has been calculated, to tune the network for the input data set. To extract the area of interest, we used the idea presented in [22]. That is, we calculate the inner product of the weight vector w and the pixel feature vectors (Figure 1). This way, the purple area of the original image will have the highest brightness intensity, whereas the rest of the image will darken.

The Gram-Schmidt process takes a finite linearly independent set *S* = {*v*_1_, ⋯, *v*_*k*_} for *k* < = *n*  and will generate an orthogonal set *S*′ = {*u*_1_, ⋯, *u*_*k*_} to span the same *k*-dimensional subspace of *R*^*n*^ as *S*. To do that, a projection operation is defined as follows:

(1) $$\begin{array}{c} {\text{proj}}_{u}^{v}=\frac{<u,v>}{<u,u>}u=<u,v>\frac{u}{<u,u>}, \end{array}$$

where <*u*, *v*> represents the inner product of operator *v* on vector u.

Given this definition, the Gram-Schmidt orthogonality method will be as follows [19]:

(2) $$\begin{array}{c} u_{1}=v_{1},\\ e_{1}=\frac{u_{1}}{\left\|u_{1}\right\|},\\ u_{2}=v_{2}-{\text{proj}}_{u_{1}}^{v_{2}},\\ e_{2}=\frac{u_{2}}{\left\|u_{2}\right\|},\\ u_{3}=v_{3}-{\text{proj}}_{u_{1}}^{v_{2}}-{\text{proj}}_{u_{2}}^{v_{3}},\\ e_{3}=\frac{u_{3}}{\left\|u_{3}\right\|},\\ u_{k}=v_{k}-\overset{k-1}{\underset{j=1}{\sum }}{\text{proj}}_{u_{j}}^{v_{k}},\\ e_{k}=\frac{u_{k}}{\left\|u_{k}\right\|}. \end{array}$$

Using this method, the w_k_ vector will be used for the set *S* = {*v*_1_, ⋯, *v*_*n*_}. Subsequently, the maximum projection on *v*_*k*_ and orthogonal to other vectors in the set is calculated as below:

(3) $$\begin{array}{c} w_{k}=v_{k}-\overset{k-1}{\underset{j=1}{\sum }}{\text{proj}}_{v_{j}}^{v_{k}}. \end{array}$$

Eventually, we can do the segmentation based on appropriate thresholds that are chosen with respect to the histogram of the result. Given that the platelet areas are smaller than the nucleus, we can remove the small pieces and the remaining part will only include the nucleus. To eliminate the effect of the color difference and the nucleus illumination intensity between image samples, three different weighting vectors are calculated for each image. Eventually, we will apply the “AND” reasoned action on the three resulting images to get the segmentation phase results. This process is illustrated in Figure 2.

### 3.2. Classification

#### 3.2.1. Scale-Invariant Feature Transform

Scale-Invariant Feature Transform (SIFT) feature detection has been used for feature extraction [23]. SIFT is based on the image gradients and is invariant to scaling and rotation [24]. It is rotation-invariant, which means even if the image is rotated, we can achieve the same result. It is scale-invariant which means changing the image scale will not affect the results. In addition, this method shows a high degree of resistance to other complex forms of transformation and illumination changes. SIFT extracts key points and feature vectors in three steps, presented in the following section [23].

**Step 1 .**

At this step, the incoming image is alternately convolved by Gaussian functions to obtain the smoothed samples of the original images. Then, the smoothed images are subtracted from each other to get the images of Difference of Gaussians (DOG).

**Step 2 .**

Next, the resulting DOG images are examined, and the maximum and minimum local points are selected as the key point. The maximum and minimum local points are the points that have the maximum or minimum values in both dimensions and scales compared to their neighbours. This feature ensures that the key points and the extracted feature vector remain invariant to the scale changes.

**Step 3 .**

Once the key points and the scales of each point are calculated in Step 1 and Step 2, the feature vectors for each key point will be calculated. First, the gradient image is calculated, which will be used to extract the key points. Subsequently, the direction of the region around the central pixel will be set on the gradient rotation of the central pixel. At this point, the gradient image is sampled for the 16∗16 regions around the central pixel of the gradient rotation. This step ensures that the extracted feature vector is invariant to rotation.

Next, the samples in a region are quantized in 8 main directions. The 16 × 16 region around the central pixel is divided into 16 regions of 4 × 4, and the histogram of gradient direction is calculated in each of these regions. Eventually, these sixteen 8-dimensional histograms form the final 128-dimensional feature vector [24].

### 3.3. Convolutional Neural Networks

In natural images, the values of pixels in a spatial neighbourhood have a high spatial dependency on each other and this dependence is independent from the neighbourhood location in the image [25]. To keep these dependencies and also to make the model invariant to spatial transformation, a convolutional neural network convolves a set of filters (*F* = {*f*_1_, *f*_2_, ⋯, *f*_*Nk*_}) on the input image and will result in the two-dimensional named as *z* in the following equation:

(4) $$\begin{array}{c} z=f_{k}*x. \end{array}$$

These filters are learned from the input data and their gradients using a back propagation algorithm. To calculate the feature map units, the convolutional filters are transmitted through a nonlinear active function such as sigmoid function or Rectified Linear Unit function. Subsequently, a pooling layer is applied on the output of the feature map units, to make it invariant to the transmissions. Pooling action *P* could be done using maximizing or averaging of feature map unities of the neighbourhood *G*:

(5) $$\begin{array}{c} P_{G}=\max_{i\in G}h_{i}. \end{array}$$

For the pooling phase, we used the maximum pooling method. This technique is used more often for the pooling phase as it takes care of negative values and does not blur the output units [26]. The result of the pooling layer will be sent to a regular fully connected network. In the last layer (the output layer), softmax activation is often used; however, in our work, we used the WTPSSR method instead of softmax function. The WTPTSSR method is a sparse method that will be described in detail in the next section. Subsequently, the whole network is trained using back propagation of the network error, which is calculated based on crossentropy of the last layer output.

(6) $$\begin{array}{c} c=-\overset{N_{c}}{\underset{c}{\sum }}y_{c}\text{loglog }\left(\hat{y_{c}}\right). \end{array}$$

The convolution network considered in this paper has the convolution layer and two max-pooling layers. Weight filters in the convolution layers are 3∗3, and zero padding is not considered in the layers.

### 3.4. Weighted Two-Phase Test Sample Sparse Representation

The weighted two-phase test sample sparse representation method (WTPTSSR) is an improvement of the method two-phase test sample representation (TPTSR) method [7]. The TPTSR method represents the test samples as a linear combination of the training samples. It then calculates the *M* nearest neighbours for each test sample based on the training samples that are most appropriate for the corresponding test sample. However, this method loses the local information, while in a lot of cases, locality is very important and holds a high recognition ratio [4]. The WTPTSSR method was presented to address this problem [27, 28]. WTPTSSR is identical to TPTSR, except that it adds locality on the *l*_2_ regularization. The steps of the WTPTSSR methods are as follows:

1. Input: *A* ∈ *R*^*m*×*N*^  training sample matrix, where *N* is the number of training samples and *m* is the number of features of each sample, and *y* ∈ *R*^*m*×1^ is the pilot sample
2. Columns *A* and *Y* are normalized to have normalized *l*_2_ norms
3. The *M* nearest neighbours for test samples are determined based on the equation below:

(7) $$\begin{array}{c} X={\left(A^{T}*A+t*W^{T}*W\right)}^{-1}*A^{T}*y, \end{array}$$

where W is a diagonal matrix and a local adaptor that penalties the distance between *y* and each pilot sample and is calculated as follows [29]:

(8) $$\begin{array}{c} W=\mathrm{diag}\left(\left[\text{dist}\left(y,a_{1}\right),\text{dist}\left(y,a_{2}\right),\cdots \text{dist}\left(y,a_{n}\right)\right]\right)\\ \text{dist}\left(y,a_{1}\right)={\left|\left|y-a_{i}\right|\right|}^{k}, \end{array}$$

where *k* is the local adaptor parameter. Note that if *k* = 0, the method will be transformed to TPTSSR. Then, the following equation will be calculated for all the training samples:

(9) $$\begin{array}{c} \text{co}{\text{n}}_{i}={\left|\left|y-a_{i}x_{i}\right|\right|}_{2}. \end{array}$$

Subsequently, *M* pilot samples with the lowest con_*i*_  value will be selected and construct matrix $\underline{A}.$

(4) In the next step, we will solve the linear equation (10), to calculate linear combination of the *M* training samples:

(10) $$\begin{array}{c} \underline{X}={\left({\underline{A}}^{T}\underline{A}+\gamma I\right)}^{-1}\;{\underline{A}}^{T}\;y, \end{array}$$

where *γ* is a positive constant and *I* is the identity matrix

Since each of the *M* selected samples belongs to the same class, the degree of collaboration between each class needs to be determined [30]. Assume that *t*_*i*_  is a sample of the *i*^th^ class represented by *a*_1_^*i*^, *a*_2_^*i*^, ⋯, *a*_*ti*_^*i*^. Using the following equation, we will examine the degree of collaboration between training samples of the *i*_th_ class in representing *y* pilot sample:

(11) $$\begin{array}{c} \text{co}{\text{n}}_{i}={\left|\left|y-\overset{t_{i}}{\underset{j=1}{\sum }}a_{j}^{i}\;x_{j}^{i}\right|\right|}_{2}. \end{array}$$

(5) Note that smaller con_*i*_ represents a greater contribution to the test sample. Therefore, the class of pilot sample *y* is determined as the class that gives the lowest value of collaboration

In the next section, we will present how our model worked on LISC and WBCis databases. We will also compare our model with four other baseline methods.

## 4. Results and Experiments

### 4.1. Segmentation Results

To assess the segmentation, we compare the similarity between manual and automatic segmentation. Higher similarity metric indicates more accurate segmentation. Similarity is calculated using the below equation:

(12) $$\begin{array}{c} T_{S}=\frac{A_{\text{Automatic}}U\;A_{\text{Manual}}}{\max\left(A_{\text{Automatic}},A_{\text{Manual}}\right)}\times 100, \end{array}$$

where *A*_Automatic_ is the area of the automated segmented core and *A*_Manual_ is the area of the manually segmented core.

### 4.2. RDE Criterion

The relative distance error criterion (RDE) is used to assess the extracted segments [26, 31]. Assume that *e*_1_, *e*_2_, ⋯.*e*_*n*_*T*__ are the *E* pixels and *t*_1_, *t*_2_, ⋯.*t*_*n*_*T*__are the *T* pixels, where *E* is the boundary of the image obtained from automated segmentation and *T* is the boundary of the image from manual segmentation. *n*_*E*_ and *n*_*T*_ are the number of segmented pixels in *E* and *T* boundaries, respectively. With these assumptions, RDE is defined according to the following equation:

(13) $$\begin{array}{c} \text{RDE}=\frac{1}{2}\left(\sqrt{\frac{1}{n_{E}}\overset{n_{E}}{\underset{i=1}{\sum }}d_{e_{i}}^{2}}+\sqrt{\frac{1}{n_{t}}\overset{n_{t}}{\underset{j=1}{\sum }}d_{t_{j}}^{2}}\right), \end{array}$$

where **d**_**t**_**j**__ and **d**_**e**_**j**__ parameters are defined based on equation (14), and **distance**(**e**_**i**_, **t**_**j**_) indicates the Euclidean distance between **e**_**i**_ and **t**_**j**_.

(14) $$\begin{array}{c} d_{e_{i}}=\min\left\{\text{distance}\left(e_{i},t_{j}\right)\;|\;j=1,2,\cdots n_{t}\right\}. \end{array}$$

### 4.3. OR, UR, and ER Criteria

**Q**_**p**_ indicates the number of pixels result from the manual segmentation that are not found in the automatic segmentation.  **U**_**P**_ represents the number of pixels that result from automated segmentation and are not found in the manual segmentation. **D**_**P**_ represents the number of pixels in the manually segmented object.

The OR, UR, and ER criteria, which, respectively, indicate oversegmentation, subsegmentation, and error ratio, are calculated according to equations (15), (16), and (17) [3, 13, 32, 33].

(15) $$\begin{array}{c} \text{OR}=\frac{Q_{p}}{U_{P}+D_{P}}, \end{array}$$

(16) $$\begin{array}{c} \text{UR}=\frac{U_{p}}{U_{P}+D_{P}}, \end{array}$$

(17) $$\begin{array}{c} \text{ER}=\frac{Q_{p}+U_{P}}{D_{P}}. \end{array}$$

Table 1 illustrates the numerical results of the proposed method for nucleus segmentation in comparison with the methods proposed in [16, 34]. As mentioned earlier, in LISC (Leukocyte Images for Segmentation and Classification) and WBCis (Wight Blood Cell Images for Segmentation) databases, the evaluation parameters are only calculated for white blood cells.

### 4.4. Classification Results

We used 260 samples of images containing 720 × 576 pixels, all of which are colored images, to detect blood cells that contain 5 different classes. In Table 1, the results of the proposed procedure are applied to 260 white cell images such as neutrophil, basophil, monocyte, eosinophil, and lymphocyte. Tables 2 and 3 are the confusion matrix where HoG descriptor and SIFT are used along with CNN to extract features, respectively. In Table 4, we compare the accuracy of the proposed method against four baseline models. In Table 5, we compare how different classification techniques, namely, SVM, WTPSSR, and distance classification, perform. Note that the same feature extraction method (the combination of CNN and SIFT) is used for this comparison.

## 5. Conclusion

Infection diseases remain a major public health issue globally. One of the effective ways to detect several life-threatening infectious diseases is using white blood cells. In this paper, we present an approach to detect different types of white blood cells in microscopic images. We used the Gram-Schmidt process for the segmentation step, and for the classification, we used the Scale-Invariant Feature Transform (SIFT) technique along with a convolutional deep neural network. In the classification phase, instead of using a softmax classification method, we utilized a sparse method which improved accuracy of our model to 97.14%. While our work provides promising results, there are some areas for further improvement that future research should explore. The first limitation of our work, like many other researches in this domain, is lack of a benchmark to evaluate and compare our results. Future research should create a benchmark for this domain and analyse how different methods would work in a single data set comparatively. Second, we did not have access to a large enough data set. Increasing the data sample size as well as the variety of the sample images could also greatly increase the accuracy and generalizability of the model. To increase the data set size and variety with the aim to increase the data independency and the classification accuracy, one potential solution would be to collect databases available in different health centres. Creating such a data set as the benchmark in this domain could be a very big step towards developing methods with higher accuracy and, more importantly, will improve the generalizability of the findings. Lastly, to apply our proposed model on a more complex data set, we can enhance the deep convolutional neural network by increasing the number of layers and the dimension of each layer to meet the complexity of a more complicated system.

## Figures and Tables

**Figure 1:** The relationship between the vector w_3_ and the vectors v_1_, v_2_, and v_3_ in the three-dimensional space.

**Figure 2:** Segmentation of white cells using the Gram-Schmidt algorithm.

**Table 1:** Numerical results of core segmentation.

Evaluation metrics	Hamghalam et al. [16]		Salem [34]		The proposed method	
	LISC data set	Sharks WBCis data set	LISC data set	Sharks WBCis data set	LISC data set	Sharks WBCis data set
*T*_*s*_	93.20	89.64	87.9	91.3	96.49	97.33
RDE	2.73	4.54	5.3	3.87	1.98	1.49
OR	0.076	0.084	0.103	0.066	0.062	0.052
UR	0.081	0.083	0.089	0.071	0.071	0.065
ER	0.179	0.194	0.24	0.156	0.128	0.134

**Table 2:** The confusion matrix when HoG descriptor is applied.

Predicted class	True class					
	Basophil	Eosinophil	Lymphocyte	Monocytes	Neutrophil	Accuracy
Basophil	45	4	0	5	1	81%
Eosinophil	5	24	1	7	2	61%
Lymphocyte	1	2	56	2	0	91%
Monocytes	13	9	2	22	2	45%
Neutrophil	0	2	0	1	54	94%

**Table 3:** The confusion matrix when SIFT and CNN descriptors are applied.

Predicted class	True class					
	Basophil	Eosinophil	Lymphocyte	Monocytes	Neutrophil	Accuracy
Basophil	53	0	2	0	0	81%
Eosinophil	0	35	2	2	0	61%
Lymphocyte	0	1	58	1	1	91%
Monocytes	0	2	3	42	2	45%
Neutrophil	0	2	0	1	54	94%

**Table 4:** Comparing the accuracy of the proposed method in detecting the white blood cells with four baseline methods.

Reference	Segmentation method	Classification method	Sample size	Accuracy
The proposed method	Gram-Schmidt orthogonalization	WTPSSR	260	97.14%
The proposed model by Rezatofighi et al. [17]	Gram-Schmidt orthogonalization and snake	SVM	400	86.10%
The proposed model by Zhang et al. [26]	Histogram threshold	Distance classifier	199	92.46%
The proposed model by Balki et al. [6]	Entropy threshold and iterative threshold	Distance classifier	71	90.14%
The proposed model by Horne et al. [2]	Gram-Schmidt orthogonalization and snake	LVQ	400	94.10%

**Table 5:** Comparing the accuracy of the proposed approach when using different classification methods (the segmentation is done using SIFT and convolutional deep neural network across these models).

Feature extraction method	Classification method	Sample size	Accuracy
CNN + SIFT	WTPSSR	260	97.14%
CNN + SIFT	SVM	260	78.5%
CNN + SIFT	Distance classifier	260	81.2%

## Data Availability

The image data used to support the findings of this study have been deposited in the WBCis repository (https://github.com/zxaoyou/segmentation_WBC).
